# VGG-UNet/VGG-SegNet Supported Automatic Segmentation of Endoplasmic Reticulum Network in Fluorescence Microscopy Images

**DOI:** 10.1155/2022/7733860

**Published:** 2022-06-08

**Authors:** Jesline Daniel, J. T. Anita Rose, F. Sangeetha Francelin Vinnarasi, Venkatesan Rajinikanth

**Affiliations:** ^1^Department of Computer Science and Engineering, St. Joseph's College of Engineering, OMR, Chennai, 600 119 Tamil Nadu, India; ^2^Department of Electronics and Instrumentation Engineering, St. Joseph's College of Engineering, OMR, Chennai, 600 119 Tamil Nadu, India

## Abstract

This research work aims to implement an automated segmentation process to extract the endoplasmic reticulum (ER) network in fluorescence microscopy images (FMI) using pretrained convolutional neural network (CNN). The threshold level of the raw FMT is complex, and extraction of the ER network is a challenging task. Hence, an image conversion procedure is initially employed to reduce its complexity. This work employed the pretrained CNN schemes, such as VGG-UNet and VGG-SegNet, to mine the ER network from the chosen FMI test images. The proposed ER segmentation pipeline consists of the following phases; (i) clinical image collection, 16-bit to 8-bit conversion and resizing; (ii) implementation of pretrained VGG-UNet and VGG-SegNet; (iii) extraction of the binary form of ER network; (iv) comparing the mined ER with ground-truth; and (v) computation of image measures and validation. The considered FMI dataset consists of 223 test images, and image augmentation is then implemented to increase these images. The result of this scheme is then confirmed against other CNN methods, such as U-Net, SegNet, and Res-UNet. The experimental outcome confirms a segmentation accuracy of >98% with VGG-UNet and VGG-SegNet. The results of this research authenticate that the proposed pipeline can be considered to examine the clinical-grade FMI.

## 1. Introduction

Artificial intelligence (AI) techniques are widely adopted in various engineering and scientific domains to obtain the finest possible solutions for a considerable number of problems. For example, AI-supported medical data assessment is one of the vital research fields. Therefore, a chosen scheme is employed to examine the information collected from hospitals and scan centers.

Typically, medical data includes the information collected from patients, such as personal data, diagnostic information, and collected biosignals and bioimages [1–3]. Assessment of medical data collected from the patient is essential during diagnosis, treatment execution, and monitoring of the recovery rate.

The literature confirms that various traditional and machine-learning (ML) procedures are employed to examine a variety of medical data with improved accuracy [4, 5]. Along with the ML schemes, deep learning (DL) procedures are also widely employed to examine various medical data to get a better diagnosis [6, 7]. The DL scheme works well on various medical databases available in the form of features, signals, and images. Therefore, it helps to achieve a superior result compared to other techniques. Most of the earlier works considered the pretrained DL procedure because of its superior result. The conventional and modified forms of the DL techniques are employed in segmentation and classification tasks [8–10].

In this work, the fluorescence microscopy image (FMI) database available in [11] is considered for the assessment. This dataset consists of the endoplasmic reticulum (ER) network image, and the study of the structural information plays a vital role in mediating cell condition assessment. Pricewise segmentation of this network is essential for evaluating the morphology needed to support the disease diagnosis and drug discovery functions. In the human cells, the ER network forms an energetic construction that supports the following functions in the cell, including calcium storage, protein synthesis, and lipid metabolism. Therefore, the segmentation and examination of ER network structure are essential in the medical domain to assess the cell's complete information and protein structure. This information can be found in [12, 13].

The extraction of ER network from the FMI is achieved using the CNN approach, and in this work, novel VGG-UNet and VGG-SegNet are enhanced with the VGG19 model. The proposed scheme is tested and validated on the benchmark FMI dataset. This dataset consists of 223 images, data augmentation is implemented to increase the image dataset to 2007 images, and each image is resized to 224 × 224 × 1 pixels. This image is then considered for testing and validating the ER network segmentation performance of the CNN technique, and the investigation is implemented using MATLAB®. A detailed comparative assessment of CNN schemes, such as U-Net, SegNet, Res-UNet, VGG-UNet, and VGG-SegNet, is presented. The segmented ER network is then compared against the ground truth (GT) available in the database, and the necessary image measures are computed. The experimental proposed investigation with the proposed schemes helped achieve a segmentation accuracy of >98%. This research confirmed that the outcome of VGG-SegNet is better than other schemes considered in this work. This work was also tested on the version of the FMI dataset existing in [11] and achieved a better result. This confirms that the proposed scheme is efficient in examining the FMI. In the future, it can be considered to evaluate the clinical-grade ER network evaluation task using the FMI.

The main contributions of this study are as follows:

- The complexity of the dataset is addressed, and to reduce the complexity, a 16-bit to 8-bit conversion is employed
- The recent CNN segmentation schemes such as VGG-UNet and VGG-SegNet are implemented to examine the fluorescence microscopy images
- Comparative analysis between the commonly considered CNN segmentation schemes is presented

Other sections of this research are organized as follows: Section 2 presents earlier works on FMI, Section 3 shows the methodology employed, and Sections 4 and 5 discuss the results and conclusions of the present research, respectively.

## 2. Related Earlier Research

The assessment of ER network morphology is a clinically significant task during the disease diagnosis and drug discovery process. Therefore, this assessment is performed to examine the cell and its related information, and in the literature, the researchers discuss several ER network examination methods.

Usaj et al. [14] discussed single-cell image-supported morphology assessment to detect the cell-to-cell variability of the internal structures. Abrisch et al. [15] presented a study regarding mitochondrial morphology regulation based on fission/fusion procedures converging to ER network. Silva et al. [16] discussed various procedures to be adopted to study the cell signaling process during cancer and neurodegenerative disorder conditions. Powers et al. [17] discuss a detailed assessment of the tubular ER network's reconstruction process.

The image processing supported cell image assessment is also widely discussed to examine the cell condition during normal and disease conditions. The research of Heinrich et al. [18] presented an automated segmentation procedure to extract the cell organelle from volumetric electron microscopy images. Chen et al. [19] discussed a novel three-dimensional residual channel attention procedure to improve the visibility of FMI. Shamir [20] presented low-level picture descriptors to support the computer-based FMI examination. Pécot et al. [21] presented a conditional random field technique-based segmentation and fluorescence estimation procedure to examine the live cell. Tahir [22] presented a detailed assessment of the morphological structure of protein images recorded using FMI. This work implemented gray level cooccurrence matrix (GLCM) technique to assess the FMI pictures. Zhang and Zhao [23] proposed a CNN scheme called CapsNet to evaluate the FMI database to classify 2D HeLa cells. Moen et al. [24] presented a detailed assessment of cellular images using a deep learning scheme. Mabaso et al. [25] present a detailed review of the assessment and segmentation of FMI.

Extracting the EM network from FMI is a complex task and achieving better segmentation accuracy is also challenging. Hence, CNN-supported segmentation is employed to extract and evaluate the ER network from FMI with better segmentation accuracy.

## 3. Methodology

This part of the work demonstrates the methodology employed to mine the ER network using the CNN scheme.

Figure 1 depicts the architecture employed in this research work to examine the FMI database. Initially, the complex FMI is collected from the dataset. The collected FMI has a complex threshold level, and its complexity is initially reduced using an image conversion process that converts the tagged image file (.tif) format into a bitmap (.bmp) with a chosen threshold of 256 and it is resized to 224 × 224 × 1 pixels. Next, image augmentation is employed to increase the number of test images, and the augmented image is then considered to train and validate the performance of the CNN scheme. After excellent training, the segmentation performance is tested, and the extracted ER network section is then compared with the GT image. Finally, based on the attained image performance, the advantage of this proposal is confirmed.

### 3.1. Image Database

This work considered the ER network FMI dataset [11] for assessment, and this dataset is formed with the help of cultured live cells; recorded with the help of spinning disk confocal microscopy (SDCM).

The recorded ER network was obtained from cells labelled with Green Fluorescent Protein (GFP), fused sec61*β*, and cultivated on MatTek cover glass dishes to 60% confluence. Pictures were collected using a 100 × 1.45 − N.A. oil W.D. 0.13 mm objective on a TI2-E reversed microscope associated with a 488 nm 150 mW laser of 4 laser combiner units (Axxis), a CSU-W1 spinning disk scan head (Yokogawa), and a 95BSI sCMOS camera focused by Nikon elements software (Nikon). This imagery is then collected as patches, and every picture is available with its G.T. image. These images were clustered into two categories: FMI version 1 (FMI1) and version 2 (FMI2), and in this study, the proposed versions were separately tested and validated. FMI1 consists of 223 test images in the chosen database, and FMI2 is associated with 175 images.

The significant complexity of this dataset is that every image is registered as a 16-bit image which exhibits a complex threshold value, and it needs a 16-bit to 8-bit conversion to support the computerized evaluation. In this work, the conversion of 16-bit to 8-bit conversion is initially performed to reduce the complexity, and the converted image is then considered for the examination. The conversion of 16-bit to 8-bit is achieved using the MATLAB command

(1) $$\begin{array}{c} 8\text{bit image}=\text{Unit}8*\left(\frac{16\text{bit image}}{256}\right). \end{array}$$

8bit image = Unit8∗(16bit image/256).  Figure 2(a) depicts the sample test image and its histogram for 16-bit and 8-bit cases as in Figures 2(b) and 2(c), respectively.

The image values are then increased using the image augmentation (picture rotation by 0 < *θ* < ±60^o^ insteps of 15^o^) process, and this helped to achieve an increase in image number to 2007 for FMI1. Figures 3 and 4 present the sample test images and augmented images considered in this research work.

### 3.2. Proposed CNN Scheme

In this research, the CNN segmentation methods, such as UNet [26] and SegNet [27], were improved using the VGG19 scheme. The earlier versions of CNN segmentation schemes are available along with VGG11 or VGG16, and these approaches have already confirmed their eminence in a class of medical images with gray/RGB scales. In this work, the conventional CNN segmentation procedures were improved by considering the VGG19 as the encoder and its inverse operation as the decoder section. The proposed encoder-decoder section was then trained to extract the ER network from the test images with better accuracy using a SoftMax classifier unit. The architecture of the VGG-UNet and VGG-SegNet is depicted in Figures 5 and 6, respectively. The necessary information on VGG-UNet and VGG-SegNet can be found in [28–32].

### 3.3. Pretraining and Segmentation

The considered CNN segmentation models were initially trained using the test/GT images to learn about the ER network, which is to be extracted from the FMI. Initially, the performances of the CNN models were tuned using optimizers, such as ADAM and stochastic gradient descent (SGD) with various batch sizes, such as 4, 8, 16, and 32 with a learning rate = 1*e* − 5, dropout rate = 20%, number of iterations = 5000, and number of epochs = 50. The initial approach helped get a better learning rate (better accuracy with lesser dice loss) when the ADAM optimizer was used with a batch size of 8. This process is repeated until a training accuracy of >95% is achieved, and the sample result achieved during this process can be found in Figure 7.

The experimental investigation is repeated using the Python®, and the attained results are presented in Figure 8.  Figure 8(a) depicts the images considered to train and validate the U-Net, and Figure 8(b) depicts the performance of the considered scheme for 100 epochs (*x* axis). Figure 8(b) confirms that the training of this scheme saturates before 50 epochs. This confirms that the pretrained scheme needs only minimum epochs to learn and extract the essential section from the considered test images. A similar result is achieved for other schemes considered in this study. This confirms that the pretrained CNN segmentation works similar when implemented with MATLAB® as well as Python®.

### 3.4. Performance Validation

The overall merit of the CNN image segmentation scheme depends on the performance values computed during the comparison of extracted ER and GT. In this work, the necessary values were computed based on the attained values of true positive (TP), true negative (TN), false positive (FP), and false negative (FN). From these values, other measures, such as Jaccard Index (JA), Dice coefficient (DI), accuracy (AC), precision (PR), sensitivity (SE), specificity (SP), *F*1-score (F1), and negative predictive value (NPV) were derived.

The representations of these values are presented in Eqs. (2) to (8) [33–39]:

(2) $$\begin{array}{c} \text{JA}=\frac{\text{TP}}{\text{TP}+\text{FP}+\text{FN}}, \end{array}$$

(3) $$\begin{array}{c} \text{AC}=\frac{\text{TP}+\text{TN}}{\text{TP}+\text{TN}+\text{FP}+\text{FN}}, \end{array}$$

(4) $$\begin{array}{c} \text{PR}=\frac{\text{TP}}{\text{TP}+\text{FP}}, \end{array}$$

(5) $$\begin{array}{c} \text{SE}=\frac{\text{TP}}{\text{TP}+\text{FN}}, \end{array}$$

(6) $$\begin{array}{c} \text{SP}=\frac{\text{TN}}{\text{TN}+\text{FP}}, \end{array}$$

(7) $$\begin{array}{c} \text{DI}=F1=\frac{2\text{TP}}{2\text{TP}+\text{FN}+\text{FP}}, \end{array}$$

(8) $$\begin{array}{c} \text{NPV}=\frac{\text{TN}}{\text{TN}+\text{FN}}. \end{array}$$

## 4. Results and Discussion

This part of work demonstrates the results achieved on a workstation; Intel i7 2.9 GHz processor with 20 GB RAM and 4 GB VRAM equipped with MATLAB®.

Initially, the pretrained U-Net is employed to segment the ER network from the FMI1 dataset. The considered CNN scheme is trained using the resized and augmented test images, this training process is continued until it achieves a training accuracy of >95%, and other procedures followed in this process are discussed in Subsection 3.3. When the CNN model is completely trained and achieved the required accuracy, then, 50 numbers of test images from FMI1 and FMI2 dataset are considered to validate the segmentation performance of the U-Net. After obtaining the necessary results, a similar procedure is then followed with SegNet, Res-UNet, VGG-UNet, and VGG-SegNet, and the results are recorded.

The result achieved at various layers of the VGG-UNet is shown in Figure 9.  Figure 9(a) depicts the various layer results of encoder section; Figure 9(b) depicts the final convolution layer outcome of decoder, Figures 9(c) and 9(d) depict the outcome of SoftMax and the binary form of the extracted ER network, respectively.

Every CNN scheme is trained using the FMI1 database (original and augmented images of data size 2007 numbers), and after the training, the segmentation performance is individually validated. The segmentation outcome achieved for a sample test image is depicted in Figure 10.  Figure 10(a) shows the GT, and Figures 10(b) to 10(f) presents the results of the CNN scheme. After collecting the binary form of the ER network, a relative assessment with GT is performed, and the obtained image measures are presented in Tables 1 and 2.  Table 1 presents the initial measures, like JA and DI, and Table 2 presents the essential performance values.

The JA, DI, and segmentation accuracy achieved with VGG-UNet are better than other methods, and the VGG-UNet and VGG-SegNet help achieve an accuracy of >99%. Even though the individual results of U-Net, SegNet, and Res-UNet are better, the comparison confirms that the proposed scheme is superior. A glyph plot is also constructed to confirm the overall performance of the proposed CNN. This plot also confirms that the overall merit of the proposed CNN scheme is better, and VGG-SegNet helps achieve a better result than VGG-UNet.

The developed scheme is verified using 50 numbers of FMI1 and FMI2 images, and the attained results are individually recorded. Finally, the mean values of the images are computed along with their standard deviation (mean ± SD), and the results are presented in Table 3. This table confirms that the segmentation accuracy achieved with the proposed CNN scheme is better (>98%), and the result of VGG-segment is comparatively reasonable than VGG-UNet. This confirms that the proposed scheme works well on the FRI database, and in the future, it can be used to assess the clinically collected FMI available from ER network.

Figure 11 presents the glyph plot, and this confirms that the result of VGG-UNet and VGG-SegNet is better than U-Net, SegNet, and Res-UNet for the Table 2 values.  Figure 12 presents the spider plot for the overall result of Table 3, and Figures 12(a) and 12(b) confirm that the VGG-UNet and VGG-SegNet provide the better result on FMI1 and FMI2 compared to other approaches. In both cases, the overall performance of VGG-SegNet is better than VGG-UNet and other CNN schemes in this study. Automatic segmentation and evaluation of the endoplasmic reticulum network in fluorescence microscopy images is a difficult task due to the image complexity. This research confirms that the proposed CNN scheme helps extract the required sections with better accuracy. The proposed scheme can be considered to examine other complex biomedical images collected from actual clinics in the future.

## 5. Conclusion

In the medical domain assessment of ER networks, structural information is essential to support disease analysis and drug discovery operations. This research employs CNN-supported segmentation to extract the ER network from the FMI dataset. This work proposes VGG19-based CNN architectures, such as VGG-UNet and VGG-SegNet, to extract the needed information from test images. In this work, two FMI image sets (FMI1 and FMI2) are considered for the assessment, and the experimental investigation is performed in a MATLAB® environment. This work presented a detailed assessment of U-Net, SegNet, Res-UNet, and the proposed schemes. The experimental outcome of this work confirmed that the proposed CNN scheme helped get a better classification accuracy (>98%), and the VGG-SegNet offered better overall performance than other techniques. In the future, this technique can be considered to examine clinically collected FMI.

## Figures and Tables

**Figure 1:** Structure of the proposed FMI examination procedure.

**Figure 2:** Sample test image and the 16-bit and 8-bit histogram values.

**Figure 3:** Sample FMI along with the associated GT image.

**Figure 4:** Augmented FMI with 0 < *θ* < ±60^o^ insteps of 15^o^.

**Figure 5:** Proposed VGG-UNet architecture.

**Figure 6:** Proposed VGG-SegNet architecture.

**Figure 7:** Training performance of VGG-SegNet for FMI1 database.

**Figure 8:** Results achieved with U-Net implemented with PYTHON®.

**Figure 9:** Sample results achieved with VGG-UNet.

**Figure 10:** Segmentation outcome achieved with the considered CNN schemes.

**Figure 11:** Glyph plot considered assessing the overall performance.

**Figure 12:** Spider plot to compare the performance of CNN schemes.

**Table 1:** Initial performance measures achieved for the chosen FMI.

CNN scheme	TP	FN	TN	FP	JA (%)	DI (%)
U-Net	6418	669	42521	568	83.8406	91.2101
SegNet	6422	676	42496	582	83.6198	91.0793
Res-UNet	6424	692	42599	451	84.8949	91.8305
VGG-UNet	7158	3	42811	185	97.4816	98.7248
VGG-SegNet	7085	0	42811	229	96.8690	98.4096

**Table 2:** Necessary performance values computed for the chosen FMI.

CNN scheme	AC (%)	PR (%)	SE (%)	SP (%)	*F*1 (%)	NPV (%)
U-Net	97.5347	91.8695	90.5602	98.6818	91.2101	98.4510
SegNet	97.4928	91.6905	90.4762	98.6490	91.0793	98.4342
Res-UNet	97.7216	93.4400	90.2754	98.9524	91.8305	98.4015
VGG-UNet	99.6312	97.4816	100	99.5697	98.7248	100
VGG-SegNet	99.5431	99.5431	100	99.4679	98.4096	100

**Table 3:** Performance measures computed for the validation images of FMI dataset.

Database	CNN scheme	AC (%)	PR (%)	SE (%)	SP (%)	*F*1 (%)	NPV (%)
FMI1	U-Net	93.05 ± 2.17	94.16 ± 1.04	91.26 ± 1.17	95.25 ± 0.84	91.31 ± 1.71	95.37 ± 0.46
	SegNet	93.73 ± 1.52	94.28 ± 0.72	91.01 ± 2.05	95.16 ± 0.63	91.51 ± 2.05	95.26 ± 1.18
	Res-UNet	97.51 ± 0.64	96.06 ± 1.13	92.25 ± 0.84	96.28 ± 1.16	92.18 ± 1.52	96.28 ± 1.05
	VGG-UNet	98.22 ± 0.51	96.28 ± 0.55	93.18 ± 1.05	97.13 ± 1.05	95.23 ± 2.03	97.34 ± 0.28
	VGG-SegNet	98.28 ± 0.63	96.18 ± 0.81	94.13 ± 1.15	96.35 ± 2.06	96.15 ± 0.72	98.11 ± 0.14
FMI2	U-net	93.72 ± 1.74	94.84 ± 0.28	91.32 ± 2.05	96.15 ± 1.05	92.05 ± 2.05	95.32 ± 1.41
	SegNet	94.06 ± 2.08	95.19 ± 1.08	91.38 ± 1.94	95.08 ± 1.26	91.28 ± 1.44	96.17 ± 1.22
	Res-UNet	97.14 ± 1.17	95.39 ± 0.42	93.07 ± 1.05	97.22 ± 1.06	92.51 ± 2.01	95.16 ± 2.31
	VGG-UNet	98.08 ± 0.27	97.15 ± 2.05	94.27 ± 0.68	97.51 ± 0.88	96.33 ± 0.53	97.50 ± 0.68
	VGG-SegNet	98.11 ± 0.31	97.36 ± 1.26	93.91 ± 0.72	97.82 ± 0.57	97.01 ± 0.18	98.09 ± 1.13

## Data Availability

The fluorescence microscopy images considered in this research work can be accessed from https://ieee-dataport.org/documents/fluorescence-microscopy-image-datasets-deep-learning-segmentation-intracellular-orgenelle
